# Estimating the Proportion of Asymptomatic COVID-19 Cases in an Italian Region with Intermediate Incidence during the First Pandemic Wave: An Observational Retrospective Study

**DOI:** 10.1155/2022/3401566

**Published:** 2022-01-06

**Authors:** Domenico Martinelli, Francesca Fortunato, Sara Mazzilli, Lucia Bisceglia, Pier Luigi Lopalco, Rosa Prato

**Affiliations:** ^1^Policlinico Riuniti Foggia Hospital, Hygiene Unit, Department of Medical and Surgical Sciences, University of Foggia, Foggia, Italy; ^2^Department of Translational Research and New Technologies in Medicine and Surgery, University of Pisa, Pisa, Italy; ^3^Scuola Normale Superiore, Pisa, Italy; ^4^Strategic Regional Health and Social Agency of Puglia (AReSS Puglia), Bari, Italy; ^5^Department of Biological and Environmental Sciences and Technology, University of Salento, Lecce, Italy

## Abstract

Early in the COVID-19 pandemic, asymptomatic transmission represented an important challenge for controlling the spread of SARS-CoV-2 through the traditional public health strategies. Further understanding of the contribution of asymptomatic infections to SARS-CoV-2 transmission has been of crucial importance for pandemic control. We conducted a retrospective epidemiological study to characterize asymptomatic COVID-19 cases occurred in the Apulia region, Italy, during the first epidemic wave of COVID-19 outbreak (February 29-July 7, 2020). We analyzed data collected in a regional platform developed to manage surveillance activities, namely, investigation and follow-up of cases and contacts, contact tracing, and laboratory and clinical data collection. We included all asymptomatic cases that were laboratory-confirmed during the appropriate follow-up, defined as persons infected with SARS-CoV-2 who did not develop symptoms/clinical signs of the disease. Between February 29 and July 7, 2020, a total of 4,536 cases were diagnosed with COVID-19 among 193,757 tests performed. The group of persons with asymptomatic SARS-CoV-2 infection consisted of 903 cases; the asymptomatic proportion was 19.9% (95% CI: 18.8-21.1%); this decreased with increasing age (OR: 0.89, 95% CI: 0.83-0.96; *p* = 0.001), in individuals with underlying comorbidities (OR: 0.55, 95% CI: 0.41-0.73; *p* < 0.001), and in males (OR: 0.69, 95% CI: 0.54-0.87; *p* = 0.002). The median asymptomatic SARS-CoV-2 RNA positive period was 19 days (IQR: 14-31) and the cumulative proportion of persons with resolution of infection 14 days after the first positive PCR test was 74%. As the public health community is debating the question of whether asymptomatic and late spreaders could sustain virus transmission in the communities, such cases present unique opportunities to gain insight into SARS-CoV-2 adaptation to human host. This has important implications for future COVID-19 surveillance and prevention.

## 1. Introduction

SARS-CoV-2 is a novel coronavirus causing the current pandemic [1], which has resulted in millions of infections and hundreds of thousands of deaths worldwide. A total of 11,500,302 coronavirus disease 2019 (COVID-19) cases were diagnosed in the world during the initial wave of the epidemic (as of July 7, 2020). Exactly 137 days since the first confirmed COVID-19 case was announced, Italy was the eleventh most affected country, with 241,819 total cases and 34,869 deaths [2], mainly concentrated in the Northern area of the country, particularly in Lombardy, Piedmont, Emilia-Romagna, Veneto, and Liguria (80% of cases diagnosed at national level). By contrast, the COVID-19 cumulative incidence remained substantially lower in the central and southern regions [3, 4].

The clinical outcomes of SARS-CoV-2 vary from asymptomatic infection to a mild-to-severe or critical disease [5, 6].

Since COVID-19 bursts onto the global scene, asymptomatic transmission of SARS-CoV-2 has appeared as the “Achilles' heel” of COVID-19 pandemic control through the traditional public health interventions [7]. Worldwide, the proportion of asymptomatic infection could be estimated to be 10.1-23.0% of all confirmed cases before May 2020 [8]. It was reported that asymptomatic infections were more common in middle-aged individuals in Shenzhen (median age: 49 years; 30.9% between 30 and 49 years) and a few younger people in Nanjing (median age: 32.5 years) [9].

Further understanding of the transmission potential of asymptomatic individuals has been crucial to improve surveillance and containment measures and estimate the likely burden of severe disease and mortality when the virus spreads in the communities [10]. However, information on the natural history of infection with SARS-CoV-2 has yet to be fully described for quantifying the contribution of persons with asymptomatic COVID-19 infection to COVID-19 transmission [11].

Here, we conducted a retrospective epidemiological study to quantify and characterize asymptomatic COVID-19 cases occurred in the Apulia region of the southern part of Italy from February 29 to July 7, 2020.

## 2. Materials and Methods

We analyzed data collected in a regional surveillance platform (GIAVA-COVID©) developed on the basis of the Go. Data outbreak investigation tool (WHO) [12] to manage the emergency. GIAVA-COVID© included functionalities for investigation and follow-up of cases (until having two consecutive negative RT-PCR test results at least 24 hours apart) and contacts (during the 14-day isolation period), contact tracing, demographics, and laboratory and clinical data collection. The collected information included age, sex, residence location, date of disease onset, date of diagnosis, date of hospital admission, date of COVID-19, test results (positive or negative), date of death, presence of underlying diseases, case outcomes (hospitalisation, virus clearance, and death), and disease severity (mild, moderate, severe, or critical) [6]. The disease classification was duly updated according to clinical evolution of each case.

This study included all asymptomatic cases, laboratory-confirmed by RT-PCR on nasopharyngeal swabs [13] that were sampled and tested according to the Italian Ministry of Health testing policies applied during the first months of the pandemic [14]. Those included close household and nonhousehold contacts of symptomatic index cases under surveillance, healthcare professionals, and solicit testing in case of risk exposure. An asymptomatic case was defined as a person infected with SARS-CoV-2 who did not develop clinical symptoms and chest imaging findings of the disease (never symptomatic individual) [9]. The asymptomatic proportion was defined as the proportion of infected individuals who were never symptomatic for COVID-19 among the total number of infected individuals [15]. The asymptomatic SARS-CoV-2 RNA positive period was defined as the number of days between the first positive PCR test and the first of the two serial negative PCR tests.

Categorical variables were summarized as the counts and percentages in each category. Continuous variables were expressed as the medians and interquartile ranges (IQR). Kruskal-Wallis test was applied to continuous variables. Binary and multivariate logistic regression analyses were performed to evaluate whether cases' demographics and clinical characteristics were independently associated with having asymptomatic infection. Analysis was conducted with STATA/SE 15.0.

As this study constituted public health surveillance, ethical approval from institutional review board was not required. All data were provided and analyzed anonymously.

## 3. Results

Between February 29 and July 7, 2020, a total of 4,536 cases (51.1% male; median age: 56 years, IQR: 41-72; cumulative incidence: 115.5 per 100,000 inhabitants) were diagnosed with COVID-19 in the Apulia region, Italy.

The group of persons with asymptomatic SARS-CoV-2 infection consisted of 903 (53.5% female) cases among 193,757 tests performed, with median age of 50 years (IQR: 32-63). Of 335 cases for whom this information was only available, 146 (43.6%) had underlying medical conditions, the most prevalent being cardiovascular disease (24.8%), neurological diseases (6.6%), diabetes (4.2%), and chronic lung disease (3%). Comparison of demographics and clinical characteristics of asymptomatic versus symptomatic presentation following SARS-CoV-2 infection are shown in Table 1.

The asymptomatic proportion was estimated to be 19.9% (95% confidence interval (CI): 18.8-21.1%). The median asymptomatic SARS-CoV-2 RNA positive period was 19 days (IQR: 14-31), and the cumulative proportion of persons with resolution of infection 14 days after the first positive PCR test was 74% (Figure 1).

The probability of having asymptomatic infection decreased with increasing age (odds ratio for being asymptomatic with each 10-year increase in age: 0.89, 95% CI: 0.83-0.96, *p* = 0.001), in individuals with underlying diseases (OR: 0.55, 95% CI: 0.41-0.73, *p* < 0.001), and in males (OR: 0.69, 95% CI: 0.54-0.86, *p* = 0.002) (Table 1).

The risk of delayed resolution of infection increased with increasing age, with median asymptomatic SARS-CoV-2 RNA positive period increasing from 16.5 days (IQR: 14-26) in persons aged 0-9 years to 28 days (IQR: 18-40) in those aged 80-89 years (*p* < 0.001).

## 4. Discussion

After the end of the first epidemic wave of COVID-19 outbreak in Italy, we tried to estimate the proportion of people with SARS-CoV-2 who were asymptomatic. Findings from our study in the Apulia region showed that between 18.8% and 21.1% of people testing positive for SARS-CoV-2 during the appropriate follow-up actions were asymptomatic. These estimates were consistent with the pooled percentages of asymptomatic infections estimated in several systematic reviews and meta-analyses performed so far during the pandemic (Table 2).

However, the Lavezzo et al. prospective cohort study conducted in the Italian municipality of Vò reported much higher proportion of asymptomatic infections (42.5%) [22]. This difference could be explained by the fact that in our study, we analyzed a larger number of cases. Moreover, the retrospective nature of our study allowed us to exclude from the analysis the asymptomatic individuals who developed symptoms later during follow-up. In fact, presymptomatic patients are easily misclassified as asymptomatic if the follow-up is not long enough, and this may lead to overestimate the true burden of asymptomatic infection [8].

From the beginning of the pandemic of SARS-CoV-2, older age, prior illnesses, and male sex have emerged as risk factors [8]. Our results showed that asymptomatic infections were more common in young individuals without underlying diseases and among females. A meta-analysis for studies with younger COVID-19-positive populations (e.g., obstetric patients) found that in these younger populations, it appeared fewer people developed symptoms compared to older groups, during similar follow-up times [23]. In Italy, this could be attributed to an underestimation of younger COVID-19 cases in the early phase of the outbreak due to various detection policies that led to the restriction of testing with swab to mainly symptomatic cases. Following the period examined in this study, when the World Health Organization guidelines were relaxed and Italy entered the transition phase, the testing policy has been broadened to various screening programmes (e.g., ahead of hospital admission for other causes, diagnostic suspicion that emerge during clinical activities, and screening/tracing activities that emerge via planned tests of travellers returning to Italy from foreign countries with higher virus circulation, immigrants, and employees) [4]. As a result, between July and mid-August 2020, when the second wave pandemic started, it was reported that overall 76% of asymptomatic cases seen in the Apulia region were aged between 0 and 50 years (median age: 28 years). It is likely that also the difference between the medians of age of asymptomatic cases in the two consecutive periods (50 vs. 28 years) reflected the sensitivity of case finding and diagnostic protocols rather than the true disease epidemiology.

Our data showed that one in four asymptomatically infected person had a positive nucleic test result to more than four weeks after the first test (Figure 1), this may indicate that the long-term infection of SARS-CoV-2 might really do exist among asymptomatic cases. In particular, long-term carrying of the virus was more common for asymptomatic older cases than the youngest cases.

This study had two main limitations. First, in view of the reasons mentioned above, asymptomatic cases in our first outbreak cohort could have represented a peculiar, underestimated fraction of the SARS-CoV-2 asymptomatic transmission. Since the beginning of the mitigation stage in late February 2020, most Italian regions experienced a severe lack of testing material and capacity leading the Italian Ministry of Health to prioritize viral RNA testing for symptomatic people and subjects at high risk for Sars-CoV-2 infections while drastically reducing testing of the asymptomatic general population [24, 25].

Second, the peak of resolution of infection observed at 14 days (Figure 1) was an artefact of the surveillance and depended on the fact that many cases were tested at day 14 before exiting the quarantine period. Anyhow, such peak did not affect either median or Q3 value calculation that were very likely to be 19 and 31 days, respectively.

## 5. Conclusions

Identifying asymptomatic cases has been of crucial importance for SARS-Cov-2 in the subsequent outbreak phases. In Italy, the national weekly epidemiological bulletins reported that asymptomatic infections have represented an increasing fraction of the infected population over time (>50% [26]), also as a result of increased testing capacity for COVID-19. The presence of a large proportion of asymptomatic and late spreaders of the virus has continued to be a challenge for controlling the pandemic. Atripaldi et al. suggested that, in Italy, the rapid spread of the second outbreak since late August could have been linked to the circulation of asymptomatic individuals and to their consistent contribution to community transmission in post lockdown [27]. They might also be contributing substantially to building herd immunity in addition to the real-life effect of the ongoing mass vaccination campaign (including indirect protection). However, further research is required to learn more about on how the virus adapts to humans and its future management, including COVID-19 surveillance, strategic testing policies, and public health interventions.

## Figures and Tables

**Figure 1:** Asymptomatic SARS-CoV-2 RNA positive period, Apulia region, Italy, February-July 2020.

**Table 1:** Comparison of characteristics between asymptomatic and symptomatic SARS-CoV-2 infections, Apulia region, Italy, February-July 2020.

Characteristics	Asymptomatic SARS-CoV-2 infections (no. 903)		Symptomatic SARS-CoV-2 infections (no. 3,633)		Total (no. 4,536)		Logistic regression analysis					
							Binary			Multivariate		
	No.	%	No.	%	No.	%	OR	95% CI	*p*	OR	95% CI	*p*
Sex												
Female	483	53.49	1,734	47.73	2,217	48.88	Ref.			Ref.		
Male	420	46.51	1,899	52.27	2,319	51.12	0.79	0.69-0.92	0.002	0.69	0.54-0.86	0.002

Age group, years												
0-9	28	3.10	47	1.29	75	1.65	Ref.			Ref.		
10-19	53	5.87	80	2.20	133	2.93	1.11	0.62-1.99	0.721	0.89	0.83-0.96	0.001
20-29	98	10.85	284	7.82	382	8.42	0.58	0.34-0.97	0.040			
30-39	125	13.84	370	10.18	495	10.91	0.56	0.34-0.94	0.029			
40-49	137	15.17	499	13.74	636	14.02	0.46	0.28-0.76	0.003			
50-59	189	20.93	696	19.16	885	19.51	0.45	0.28-0.75	0.002			
60-69	100	11.07	560	15.41	660	14.55	0.3	0.18-0.50	<0.001			
70-79	63	6.98	436	12.00	499	11.00	0.24	0.14-0.41	<0.001			
80-89	77	8.53	467	12.85	544	11.99	0.28	0.16-0.46	<0.001			
≥90	33	3.65	194	5.34	227	5.00	0.27	0.16-0.52	<0.001			

Single comorbidities^∗^												
None	189	56.42	676	35.39	865	38.53	Ref.			Ref.		
Cardiovascular disease	83	24.78	733	38.38	816	36.35	0.41	0.37-0.54	<0.001			
Diabetes	14	4.18	244	12.77	258	11.49	0.21	0.12-0.36	<0.001			
Chronic pulmonary disease	11	3.28	232	12.15	243	10.82	0.17	0.09-0.32	<0.001			
Cancer	9	2.69	141	7.38	150	6.68	0.23	0.11-0.46	<0.001			
Neurological diseases	22	6.57	178	9.32	200	8.91	0.44	0.28-0.71	0.001			
Chronic kidney disease	3	0.90	110	5.76	113	5.03	0.1	0.03-0.31	<0.001			
Obesity	5	1.49	89	4.66	94	4.19	0.2	0.08-0.5	0.001			
Other metabolic diseases	10	2.99	58	3.04	68	3.03	0.62	0.31-1.22	0.170			
Liver disease	2	0.60	33	1.73	35	1.56	0.22	0.05-0.91	0.037			
HIV	2	0.60	26	1.36	28	1.25	0.27	0.06-1.17	0.081			
At least one comorbidity	146	43.58	1,234	64.61	1,380	61.427	0.42	0.33-0.53	<0.001	0.55	0.41-0.73	<0.001

Ref.: reference group. ^∗^2,245 cases (335 asymptomatic and 1,910 symptomatic infections) for whom the information was available.

**Table 2:** The proportion of asymptomatic SARS-CoV-2 infections reported in different systematic reviews and meta-analyses.

First author	Study period	Total SARS-CoV-2, no.	Asymptomatic SARS-CoV-2, no.	Pooled proportions
A. Kronbichlera et al. [16]	December 1, 2019 to March 29, 2020	NR	506	24.2% (SD 22.06)
J. Zhu et al. [17]	January 1 to February 28, 2020	3,062	158	11.9% (95% CI: 2.9-25.8%)
C. Chen et al. [18]	January 1 to May 13, 2020	20,152	NR	13.34% (95% CI: 10.86–16.29%)
J. He et al. [8]	Before May 20, 2020	50,155	1,430	15.6% (95% CI: 10.1-23.0%)
D. Buitrago-Garcia et al. [19]	March 25 to June 10, 2020	6,616	1,287	20% (95% CI: 17–25%)
M. Alene et al. [20]	June 1 to December 9, 2020	6,071	1,917	25% (95% CI: 16-38%)
P. Sah et al. [21]	January 1, 2020 to April 2, 2021	17,272	7,222	35.1% (95% CI: 30.7-39.9%)

NR: not reported. SD: standard deviation.

## Data Availability

The data that support the findings of this study are available from the Apulia Public Health Authority, but restrictions apply to the availability of these data, which were used under license for the current study, and so are not publicly available. Data are however available from the authors upon reasonable request and with permission of the Apulia Public Health Authority.
